The article "Artificial Intelligence Algorithm-Based MRI in the Diagnosis of Complications after Renal Transplantation" was published in 2022. Journal: Contrast Media Mol Imaging.

# Artificial Intelligence Algorithm-Based MRI in the Diagnosis of Complications after Renal Transplantation

**DOI:** 10.1155/2022/8930584

**Published:** 2022-08-16

**Authors:** Hang Liu, Liang Ren, Bohan Fan, Wei Wang, Xiaopeng Hu, Xiaodong Zhang

**Affiliations:** Department of Urology, Capital Medical University Beijing Chaoyang Hospital, Beijing 100020, China

## Abstract

This study was to explore the diagnostic value of magnetic resonance imaging (MRI) optimized by residual segmentation attention dual channel network (DRSA-U-Net) in the diagnosis of complications after renal transplantation and to provide a more effective examination method for clinic. 89 patients with renal transplantation were selected retrospectively, and all underwent MRI. The patients were divided into control group (conventional MRI image diagnosis) and observation group (MRI image diagnosis based on DRSA-U-Net). The accuracy of MRI images in the two groups was evaluated according to the comprehensive diagnostic results. The root mean square error (RMSE) and peak signal-to-noise ratio (PSNR) of DRSA-U-Net on T1WI and T2WI sequences were better than those of U-Net and dense U-Net (*P* < 0.05); comprehensive examination showed that 39 patients had obstruction between ureter and bladder anastomosis, 13 cases had rejection, 10 cases had perirenal hematoma, 5 cases had renal infarction, and 22 cases had no complications; the diagnostic sensitivity, specificity, accuracy, and consistency of the observation group were higher than those of the control group (*P* < 0.05). In the control group, the sensitivity, specificity, and accuracy in the diagnosis of complications after renal transplantation were 66.5%, 84.1%, and 78.32%, respectively; in the observation group, the sensitivity, specificity, and accuracy in the diagnosis were 67.8%, 86.7%, and 80.6%, respectively. DRSA-U-Net denoising algorithm can clearly display the information of MRI images on the kidney, ureter, and surrounding tissues, improve its diagnostic accuracy in complications after renal transplantation, and has good clinical application value.

## 1. Introduction

The development of renal transplantation has gone through a long process and has now become the first in the field of peripheral organ transplantation [1]. Transplantation is the best treatment for end-stage renal failure. However, the incidence of renal insufficiency after transplantation is still very high, and the occurrence of complications after transplantation is the main factor causing the function loss of transplanted kidney [2]. The key to improve transplant survival is early and accurate diagnosis and appropriate treatment. In recent years, with the development of imaging techniques, it is very helpful for the early diagnosis of complications after renal transplantation [3]. Complications after renal transplantation seriously affect clinical outcomes and can lead to loss of transplanted organ function and patient's death. According to the United States Joint Network for Organ Sharing, by the end of 2020, the total number of kidney transplants reached 1.3 million worldwide and approximately 160,000 in China [4].

The article "Artificial Intelligence Algorithm-Based MRI in the Diagnosis of Complications after Renal Transplantation" was published in 2022. Journal: Contrast Media Mol Imaging.

At present, the process of renal transplantation has been standardized, the new triple suppression regimen exerts the greatest immunosuppressive function with the least drug toxicity, the first-year survival rates of patients and grafts are more than 96% and 91%, respectively, and the quality of life of patients is significantly improved [5]. The reported incidence of complications in renal transplantation is 3–21%, and the incidence of vascular complications is 1.8–8.4%. It is generally believed that complications after renal transplantation can be divided into functional complications and organic complications. Therefore, surgical complications should be paid attention [6].

U-Net was proposed by Marticorena Garcia et al. [7] and named for its left-right symmetry of the network structure and resembling the letter “U.” U-Net is mainly composed of two parts: the contraction path on the left side and the expansion path on the right side. The contraction path is mainly used for feature extraction, the expansion path is mainly used to decode the feature map, and the upper sampling is used to improve the resolution of the feature map. Compared with other networks, Dense-U-Net improves network performance by reducing information loss from network depth or width and is committed to improve network performance from the perspective of feature reuse [7]. Abdominal movement is complex, and MRI is highly sensitive to movement. Therefore, abdominal MRI is more complex to perform the image acquisition and processing than other positions [8]. Like abdominal image-assisted acquisition technique commonly used, abdominal T1WI generally includes in-phase T1WI and out-of-phase T1WI. However, other sites are not so distinguished. Current deep learning-based transmodal synthesis studies of MRI basically use brain MRI data, mainly focusing on MRI, CT, and PET, while there are few transmodal synthesis studies of MRI-weighted images [9]. In the image evaluation of renal transplantation, MRI is superior to CT because of its better soft tissue resolution and no radiation injury. In addition, MRI contrast agent has no damage to the kidney, and MSCT and CTA can visually show the situation of renal transplantation. Interlayer registration of multimodal images: image synthesis usually requires registration among images, but in the actual MRI scan, due to slice thickness and scanning environment, the registration requirements are difficult to meet [10]. Although some deep learning algorithms can achieve cross-channel unregistered synthetic images, they are mainly large networks such as gallium nitride, which usually means that a large amount of data is needed to solve many parameters in the network, which is a great threat to scarce medical images [11, 12]. Transmodal image synthesis networks are usually single-channel networks synthesized by single-modal images, but some studies have demonstrated that the effect of multimodal information synthesis is much better than that of single-modal image synthesis [13]. The improved U-type residual segmentation attention dual channel network (DRSA-U-Net) strengthens the ability of the network to extract and fuse the characteristic information of multichannel images by introducing the separation attention residual module and the compression excitation attention module in U-Net. It effectively improves the effect of the network to synthesize images. Therefore, how to make full use of multimodal data information and design multichannel networks with good learning performance according to image characteristics is also a research topic.

The article "Artificial Intelligence Algorithm-Based MRI in the Diagnosis of Complications after Renal Transplantation" was published in 2022. Journal: Contrast Media Mol Imaging.

This study was aimed to explore the diagnostic value of optimized MRI based on DRSA-U-Net in the diagnosis of complications after renal transplantation and to provide a more effective examination method for clinic.

## 2. Materials and Methods

### 2.1. Subjects

In this study, 89 patients who underwent renal transplantation in hospital from March 2020 to March 2021 were included and examined by MRI. The patients received MRI at 2 weeks after operation. The patients were randomly divided into the control group (conventional MRI image diagnosis) and the observation group (MRI image diagnosis based on DRSA-U-Net). There were 59 males and 30 females, aged 27–46 years, with the mean age of 42 years. 76 transplanted kidneys were located in the right iliac fossa and 13 transplanted kidneys in the left iliac fossa; 45 developed tenderness 30 days after surgery; 37 had anuria 9 days after surgery; and 7 had postoperative fever and abdominal pain. This study approved by the ethics committee of the hospital, and the patients' families signed the consent form.

Inclusion criteria: all patients received renal transplantation; those who follow doctor's advice and actively cooperate with the treatment.

Exclusion criteria: history of contrast medium allergy; those who are allergic to the drugs used; patients with other types of serious diseases; heart, liver, spleen, and other important organ dysfunction.

The article "Artificial Intelligence Algorithm-Based MRI in the Diagnosis of Complications after Renal Transplantation" was published in 2022. Journal: Contrast Media Mol Imaging.

### 2.2. MRI Scan

1.6*T* superconducting MRI scanner was used, gradient was 32 mT/m, switching rate was 132 Tm^−1^ s^−1^, and flexible phased array circular polarization coil was used. Examination order and parameters: referring to the clinical symptoms of patients, laboratory tests, and ultrasound results, with different sequences, all patients underwent routine renal MRI and magnetic resonance urography (MRU) examination. Sequence and main parameters: axial, spin echo (SE) sequence T1WI, TR/TE was 112 ∼ 124 ms/4.85 ms; fast spin echo (FSE) sequence fat suppression T2WI, TR/TE was 2,121 ∼ 2,406 ms/132 ms; coronal TRUFI sequence, TR/TE was 5.1 ms/2.56 ms; layer thickness was 7 mm; spacing was 2.1 mm; average signal number was 2–4; and acquisition matrix was 258 × 258. T1WI without fat suppression and T2WI underwent fat suppression and nonfat suppression scanning 3 times, and field of vision (FOV) was 34 cm × 38 cm.

Renal MRU examination: single-shot fast spin-echo sequence (SSFSE), thick T2WI, TR/TE was infinite, layer thickness was 82 mm, interval was 0, FOV was 4,002 mm × 402 mm, and acquisition matrix was 314 × 258; thin T2WI, TR/TE was 1,123 ms/567 ms, flip angle was 152, layer thickness was 5 mm, interval was 0, FOV was 352 mm × 352 mm, and acquisition matrix was 258 × 158.

### 2.3. Image Segmentation by Artificial Intelligence Algorithm

In the separation attention residual module, the convolution kernel is first separated into several branches for individual learning. Then, the features learned from different branch channels are compressed and fused through the global pooling layer. Finally, the *r*-Softmax of attention mechanism is used to extract features, and the extracted features and the output of each branch are multiplied and added to obtain the feature layer with the same dimension as the input. In the parallel space channel compression and excitation module, DRSA-U-Net adds Scse module after each jump connection in U-Net to compress and excite the MRI images of T1WI and T2 downsampling weighted image. It can extract the effective information in each channel and space and enhance the learning efficiency of the network. The biggest feature of these algorithms is that the learning rate remains unchanged. Parameter update can only be achieved by gradient, and in equation (1), *U* represents the learning rate.

(1) $$\begin{array}{c} \mu =\mu -u\cdot \nabla_{\mu }J. \end{array}$$

Because of the slow calculation of this algorithm, another algorithm is proposed. The calculation speed vector of this algorithm introduces *w* as the momentum, which reflects the direction and speed of the parameters in the parameter space. *w* value is equal to the average negative gradient exponential decay, including *b* hyperparameters. The value range is [0, 1). The parameters are expressed in equation (3).

(2) $$\begin{array}{c} w=b\cdot w-u\cdot \nabla_{\mu }J, \end{array}$$

(3) $$\begin{array}{c} \mu =\mu +v. \end{array}$$

Parameter is modified in real time, and its scaling Δ*μ* equivalently achieves adaptive learning rate. The global learning rate is denoted as Ψ. The algorithm is defined by equations (4) to (6). The implementation of the algorithm can be divided into three steps: first, the second-order momentum *p* was calculated; then, the parameter variation value Δ*μ* is calculated; finally, parameter *μ* is updated. The scaling part Δ*μ* of each parameter is inversely proportional to the sum square root $\sqrt{p}$ of the square value of the historical gradient. Therefore, the parameters with large partial derivatives correspond to larger learning rate, and the parameters with small partial derivatives correspond to smaller parameters. During the training process, the learning rate is adjusted according to the parameters. The exponential decay rate factor of first-order momentum and second-order momentum is in the range of [0, 1). The algorithm takes into account the first-order and second-order derivatives and also completes the adaptive adjustment of learning rate in network training. It has high robustness to the selection of hyperparameters and is the most widely used optimized deep learning algorithm.

(4) $$\begin{array}{c} p=p+{\left(\nabla_{\mu }J\right)}^{2}, \end{array}$$

(5) $$\begin{array}{c} \Delta \mu =-\Psi \frac{1}{\sqrt{p}+\delta }\nabla_{\mu }J, \end{array}$$

(6) $$\begin{array}{c} \mu =\mu +\Delta \mu . \end{array}$$

DRSA-U-Net is based on the traditional U-Net structure. The left side is composed of three encoders. There is a 65 × 4 × 4 convolution layer before the first encoder, which extracts the input of two channels into 65 channels. The first encoder is composed of three independent note residual modules and average titer sampling. The second encoder is composed of four independent residual modules and average sampling, and its output is 65 channels. Then, the output image is sampled. The third encoder is composed of five independent note residual modules and average sampling, and there are 256 output channels. The encoder is composed of three decoders. Each decoder is composed of an interpolation module. The decoder corresponding to each encoder jumps to connect with a convolution layer. The compression module is also added to the clock excitation attention of the second and third decoding units. The interpolation module samples the image through the nearest neighbor of interpolation and extracts the compression excitation attention module of channel and spatial information. The convolution layer fuses the feature channel. The output channels behind each decoder are 129, 65, and 17. At the end of the network, the output of the network is merged into a channel through the convolution layer.  Figure 1 shows the analysis model of DRSA-U-Net network data.

The article "Artificial Intelligence Algorithm-Based MRI in the Diagnosis of Complications after Renal Transplantation" was published in 2022. Journal: Contrast Media Mol Imaging.

### 2.4. Image Analysis and Observation Indicators

The examination results of all patients were analyzed by two independent reviewers, and a consensus was reached on the controversial results after discussion. Observation: whether there was abnormal signal in the transplanted kidney, whether the boundary of renal corticomedullary was clear, whether the ureter was unobstructed, whether there was abnormal signal around the kidney, whether the transplanted renal vessels were unobstructed, and whether the cortical enhancement density was uniform.

### 2.5. Statistical Analysis

Statistics was completed using SPSS16 software. Measurement data were expressed by $\left(\bar{x}\pm s\right)$, and enumeration data were expressed by frequency or percentage (%). Kappa was used to analyze the correlation between data. *P* *<* 0.05 was considered statistically significant.

## 3. Results

### 3.1. Evaluation of MRI Image Segmentation Effect Based on Artificial Intelligence Segmentation Algorithm

The image quantification indexes of synthetic T2WI under different inputs of U-Net, Dense-U-Net, and DRSA-U-Net networks were displayed. The data were the mean value ± standard deviation of the synthetic images of all layers in the test set. When 1/4 downsampling T2WI was added to synthesize T2WI after input, the mean peak signal-to-noise ratio (PSNR) of DRSA-U-Net synthesized T2WI was enhanced by about 0.5 dB and 0.9 dB, respectively, compared with U-Net and Dense-U-Net, and the mean root mean square error (RMSE) was reduced by about 0.03 and 0.02, compared with U-Net and Dense-U-Net; when 1/8 downsampling T2WI was added to synthesize T2WI after input, the PSNR of DRSA-U-Net synthesized T2WI was enhanced by about 1.6 dB and 1.9 dB, compared with U-Net and Dense-U-Net, and the RMSE index was the same as Dense-U-Net, reduced by about 0.02 and 0.02, compared with U-Net; therefore, no matter how much downsampling rate T2WI was added to the input, the fidelity of T2WI synthesized by DRSA-U-Net was good.

The proposed DRSA-U-Net network, T2WI synthesized in the task of multimodality MRI image synthesis of abdominal T2WI, the objective image index, the visual effect of the synthesized image, or the network performance was better than the classical medical image synthesis networks U-Net and Dense-U-Net. The RMSE and PSNR of DRSA-U-Net on T1WI and T2WI were better than those of U-Net and Dense-U-Net (*P* < 0.05) (Figures 2 and 3).

The article "Artificial Intelligence Algorithm-Based MRI in the Diagnosis of Complications after Renal Transplantation" was published in 2022. Journal: Contrast Media Mol Imaging.

The T2WI synthesized by U-Net, Dense-U-Net, and DRSA-U-Net networks under different input methods was compared. The PSNR and RMSE were calculated by the current image and the real T2WI (blue box). The PSNR and RMSE of the T2WI synthesized by DRSA-U-Net were the best. In terms of visual effect, the T2WI synthesized by U-Net and Dense-U-Net, DRSA-U-Net network was very similar to the real T2WI, but the degree of ambiguity was different. In order to observe the details, the selected part of the composite image (blue box) was amplified, and the difference in detail and texture of the composite image was found. The T2WI synthesized by DRSA-U-Net network was closer to the real image, and the ambiguity was the smallest.  Figure 4 shows the results of T2WI synthesis when the three networks at 1/4 downsampling T2WI.

### 3.2. Imaging Examination

The results of comprehensive examination of 89 patients were as follows: 39 cases of hydronephrosis of the transplanted kidney, hydronephrosis of the renal pelvis of the transplanted kidney, ureteral dilatation, and obstruction at the bladder; 13 cases of blurred corticomedullary demarcation of the transplanted kidney, slightly increased signal intensity of the transplanted kidney parenchyma on T2WI, significantly increased fat suppression signal on the T2 sequence, blurred renal corticomedullary structure, and abdominal effusion, which were diagnosed as rejection; 10 cases of perirenal hematoma formation, hematoma formation around the transplanted kidney, ureteral compression, and hydronephrosis; 5 cases of vascular occlusion of the transplanted kidney, vascular occlusion, and local renal infarction 2 days after the operation. There were no complications in 22 patients (Figure 5).

### 3.3. Sensitivity, Specificity, and Accuracy Comparison

The sensitivity, specificity, and accuracy of conventional MRI images (control group) in the diagnosis of complications after renal transplantation were 66.5%, 84.1%, and 78.32%, respectively. The sensitivity, specificity, and accuracy of MRI images based on DRSA-U-Net (observation group) were 67.8%, 86.7%, and 80.6%, respectively (Figure 6).

## 4. Discussion

Rejection of the transplanted kidney is a series of cellular and fluid immune reactions of the recipient kidney to graft antigens and can occur in 91% of patients [14]. With the continuous improvement of hardware and software, MRI can provide more information on the kidney, blood vessels, ureter, and perirenal structure after renal transplantation [15]. On T1WI, the skin and medulla of the normal kidney are clearly demarcated. The disappearance of this manifestation is common in rejection or acute tubular necrosis (ATN). However, a clear boundary between the skin and medulla does not preclude rejection [16]. In 57 MRI examinations in 33 patients, it was found that 12 patients with normal renal function had well-defined renal corticomedullary borders and renal vessels entering the parenchyma after transplantation, reaching the cortex in 39%; while in 22 patients with acute or chronic rejection, the normal corticomedullary borders showed a demarcation rate of only 8.2%. The visualization rate of renal parenchymal vessels was 33%, and the visualization rate of reaching the cortex was only 8.7%. In the experiment, 13 patients showed blurred borders of the renal cortex and medulla on T1WI and increased renal signal intensity on T2WI and coronal TRUFI sequences, suggesting increased water content in the renal parenchyma, consistent with rejection. Obstruction and brain water are common rejection [17]. Uremic patients with long-term dialysis have poor physical and vascular conditions, and in the case of high-dose immunosuppressive agents, there are many complications after renal transplantation. If not treated properly, it can cause graft loss and endanger the patient's life. Although significant progress has been made in the timely detection and diagnosis of renal transplantation complications, patients still face serious posttransplantation complications, and postoperative medical and surgical complications are still important factors of morbidity and mortality [18]. Baumgartner et al. explored 56 MRI examinations of 32 patients. It was found that 11 patients with normal renal function after transplantation had clear renal cortex and medulla boundaries, and the renal blood vessels entered the parenchyma and reached the cortex in 38% of the cases. For 21 patients with acute or chronic rejection, the display rate of normal cortex and medulla boundaries was only 8%, the display rate of blood vessels in the renal parenchyma was 32%, and the renal blood vessels entered the parenchyma and reached the cortex in 8% of the cases [19]. This is related to the experimental results. Due to timely diagnosis and surgical treatment, 39 cases of hydronephrosis and dilatation were treated.

The article "Artificial Intelligence Algorithm-Based MRI in the Diagnosis of Complications after Renal Transplantation" was published in 2022. Journal: Contrast Media Mol Imaging.

There are few reports of vascular occlusion and regional renal infarction in the transplanted kidney. In the experiment, 5 patients were diagnosed with vascular occlusion and regional renal infarction by MSCTA after renal transplantation, which was confirmed by surgery.

Perirenal bleeding after renal transplantation to form a periureteral hematoma and compression of the ureter to form hydronephrosis is a rare complication that requires definitive diagnosis and urgent surgical treatment [20, 21]. The vascular empty signal of MRI can rule out venous thrombosis and provide a strong basis for the development of a safe surgical plan [22]. Based on the U-Net network, a separation attention residual module and a compression excitation attention module were introduced to improve the feature mining ability of multichannel information [23, 24]. The proposed DRSA-U-Net network-based abdominal multimodal image synthesis algorithm can obtain synthetic images very close to the real images in terms of visual effects and image accuracy. The use of synthetic images instead of real images can reduce the scanning time of abdominal MRI images and reduce the difficulty of abdominal MRI image acquisition, providing a new path for obtaining low-cost and rapid multimodality abdominal MRI images in a short time [25].

## 5. Conclusion

In conclusion, the DRSA-U-Net denoising algorithm can clearly show the information of MRI images on the kidney, ureter, and surrounding tissues and improve the diagnostic accuracy of complications after renal transplantation, which has a good clinical application value. However, there is a small sample size, and clinical trials should be conducted in multicenter hospitals with large sample size, rather than in a single area or small area. For the application of spatial information of three-dimensional data, new multimodality images with strict interlayer registration can be acquired to further verify the relationship between multilayer input and interlayer registration. Network performance needs to be validated and optimized on multiple different data sets to improve the generalization capability of the network.

## Figures and Tables

**Figure 1:** Analysis model of DRSA-U-Net network data.

**Figure 2:** Comparison of RMSE and PSNR of different networks in T1WI. (a) Synthesis of T1WI RMSE. (b) Synthesis of T1WI PSNR. ^*∗*^Compared with U-Net, *P* < 0.05.

**Figure 3:** Comparison of RMSE and PSNR of different networks in T2WI. (a) Synthesis of T2WI RMSE. (b) Synthesis of T2WI PSNR. ^*∗*^Compared with U-Net (*P* < 0.05).

**Figure 4:** T2WI synthesized by three networks at 1/4 downsampling T2WI. The blue box indicates the PSNR and RMSE calculated from the current image and the real T2WI.

**Figure 5:** Examination results of 89 patients.

**Figure 6:** Comparison of diagnostic sensitivity, specificity, and accuracy between the control group and observation group.

## Data Availability

The data used to support the findings of this study are available from the corresponding author upon request.
